# To Join or Not to Join: Decision Points Along the Pathway to Double-Strand Break Repair vs. Chromosome End Protection

**DOI:** 10.3389/fcell.2021.708763

**Published:** 2021-07-12

**Authors:** Stephanie M. Ackerson, Carlan Romney, P. Logan Schuck, Jason A. Stewart

**Affiliations:** Department of Biological Sciences, University of South Carolina, Columbia, SC, United States

**Keywords:** telomeres, double-strand break, DNA repair, homologous recombination, non-homologous end joining

## Abstract

The regulation of DNA double-strand breaks (DSBs) and telomeres are diametrically opposed in the cell. DSBs are considered one of the most deleterious forms of DNA damage and must be quickly recognized and repaired. Telomeres, on the other hand, are specialized, stable DNA ends that must be protected from recognition as DSBs to inhibit unwanted chromosome fusions. Decisions to join DNA ends, or not, are therefore critical to genome stability. Yet, the processing of telomeres and DSBs share many commonalities. Accordingly, key decision points are used to shift DNA ends toward DSB repair vs. end protection. Additionally, DSBs can be repaired by two major pathways, namely homologous recombination (HR) and non-homologous end joining (NHEJ). The choice of which repair pathway is employed is also dictated by a series of decision points that shift the break toward HR or NHEJ. In this review, we will focus on these decision points and the mechanisms that dictate end protection vs. DSB repair and DSB repair choice.

## Introduction

DNA double strand breaks (DSBs) originate from exposure to both external DNA damaging agents, such as genotoxic chemicals and ionizing radiation (IR), and endogenous sources, such replication fork collapse, reactive oxygen species and chromosome fusions (Symington and Gautier, 2011; Ceccaldi et al., 2016). DSBs can be beneficial or detrimental depending on the context. On the one hand, programmed DSBs can be beneficial to promote genome and antibody diversity in meiosis and V(D)J recombination, respectively. However, DSBs caused by DNA damage are almost always detrimental and result in deletions, translocations, and chromosome fusions, which leads to senescence, apoptosis or oncogenesis (Phillips and McKinnon, 2007; Bohgaki et al., 2010; Bunting and Nussenzweig, 2013; Rulten and Caldecott, 2013; Ghosh et al., 2018; Seol et al., 2018). To prevent such outcomes, cells activate a DNA damage response (DDR), which is predominantly mediated by the phosphatidylinositol 3-kinase-related kinase (PIKK) family members, DNA-dependent protein kinase (DNA-PK), ataxia-telangiectasia mutated (ATM), and ATM and RAD3-related (ATR) (Blackford and Jackson, 2017). These kinases signal to downstream cell cycle checkpoints and localize repair machinery to the break (Blackford and Jackson, 2017). DSBs are repaired by two major pathways, namely homologous recombination (HR) and non-homologous end joining (NHEJ) (Figure 1).

**FIGURE 1:** Overview of DSB repair pathways. Left, homologous recombination (HR) involves resection of the DNA ends by various nucleases. The ssDNA generated is then bound by RPA. Next, there is an exchange of RPA for RAD51, which facilitates the homology search and repair of the DSB. Center, for non-homologous end joining (NHEJ), the DNA ends are bound by Ku70/80 heterodimers promoting the binding of DNA-PKcs. This creates a binding platform for XRCC4, XLF, and LIG4, which facilitate ligation of the DNA ends. Right, DSBs can also be repaired by alternative-end joining (alt-EJ) or single strand annealing (SSA) pathways. These involve the use of short homologous sequences that are exposed by resection of the break. Following alignment, the DNA flaps are removed and the DNA ligated. Alt-EJ uses around 2 to 20 base pairs (bp) of homology and SSA > 25 bp to align sequences.

Homologous recombination is highly accurate and typically occurs in S/G2 phases of the cell cycle when a replicated sister chromatid is present (Burma et al., 2006; Sullivan and Bernstein, 2018). To initiate HR, the DNA ends are resected to generate long 3′ single-stranded (ss)DNA overhangs, which pair with homologous sequences. These templates are then used for DNA synthesis and repair of the break (Symington and Gautier, 2011). This process is mostly error-free, can repair protein-blocked ends and is facilitated by RAD51, a recombinase with ATPase activity which initiates strand invasion and DNA synthesis (Mehta and Haber, 2014). NHEJ, on the other hand, is fast, selective for two-ended DSBs, and often mutagenic (Ranjha et al., 2018; Stinson et al., 2020). Although NHEJ is active in all phases of the cell cycle, it occurs most frequently in G1 phase and repairs about 80% of IR-induced DSBs, making it the predominant repair pathway in mammalian cells (Burma et al., 2006; Beucher et al., 2009). To initiate NHEJ, the Ku70/80 heterodimer (hereafter referred to as Ku) and the DNA-PK catalytic subunit (DNA-PKcs) are recruited to damage sites to generate the DNA-PK holoenzyme (Gell and Jackson, 1999; Singleton et al., 1999; Jette and Lees-Miller, 2015). DNA-PK bridges the DNA ends creating a long-range synapse (Graham et al., 2016; Chen et al., 2021). Additional proteins X-Ray Repair Cross Complementing 4 (XRCC4), XRCC4-like factor (XLF) and DNA ligase 4 (LIG4) are recruited to align and ligate the DNA ends (Blackford and Jackson, 2017). To complicate matters, DSBs can also be repaired by alternative-end joining (alt-EJ; also known as DNA polymerase θ-mediated end joining) and single-strand annealing (SSA) pathways (Figure 1; McVey and Lee, 2008; Frit et al., 2014; Iliakis et al., 2015; Sallmyr and Tomkinson, 2018; Seol et al., 2018). Both pathways require some resection and utilize short regions of homology to pair the DNA ends together (Seol et al., 2018).

While DSBs must be quickly recognized and repaired to preserve genome stability, the natural chromosome ends, known as telomeres, must be protected from the DDR to prevent genome instability in the form of chromosome fusions and degradation. Telomeric DNA ranges in length from a few hundred base pairs in yeast to tens of kilobases in mammals (Blackburn, 1991; Greider, 1991). In humans, telomeres consist of short tandem 5′-TTAGGG-3′ repeats on the G-rich strand and complimentary 5′-CCCTAA-3′ repeats on the C-rich strand (Figure 2A). The G-rich strand also contains a 3′ ssDNA region referred to as the G-overhang (Makarov et al., 1997; McElligott and Wellinger, 1997). In mammals, telomeres are protected by the shelterin complex, comprised of telomere repeat-binding factors 1 and 2 (TRF1 and TRF2), repressor activator protein 1 (RAP1), TRF1-interacting nuclear factor 2 (TIN2), telomere protection protein 1 (TPP1) and protection of telomeres 1 (POT1) (Figure 2B; de Lange, 2018). Shelterin components have been identified in most eukaryotes, however, the number of known components can vary or shelterin subunits may be missing entirely, such as in *Saccharomyces cerevisiae* (de Lange, 2001, 2005). The duplex DNA is bound by TRF1 and TRF2/RAP1 whereas the G-overhang region is protected by POT1, which complexes with TPP1. Unlike humans, which contain a single POT1 gene, mice have two separate POT1 genes, POT1a and POT1b. These genes are proposed to have arisen from a duplication event (Hockemeyer et al., 2006). While clearly orthologous, POT1a and POT1b have evolved to provide slightly different activities in telomere protection (Hockemeyer et al., 2006; Wu et al., 2006; Palm et al., 2009; Kibe et al., 2010). POT1a has been shown to repress the DDR while POT1b controls 5′-end resection (Hockemeyer et al., 2006; Wu et al., 2006; Kibe et al., 2010). TPP1 interacts with TIN2 to bridge the double-stranded and single-stranded bound portions of shelterin. As described in more detail below, shelterin plays a critical role in telomere end protection and preventing the recognition of telomeres as DNA damage.

**FIGURE 2:** Overview of telomeres. **(A)** Telomeres consist of a repetitive DNA sequence that forms a duplex DNA region and a 3′ G-rich ssDNA overhang (C-strand, red: G-strand, blue). **(B)** Telomeres are bound by the shelterin complex (TRF1-TRF2-RAP1-TIN2-TPP1-POT1) and the CST complex (CTC1-STN1-TEN1), which aid in telomere maintenance. **(C)** Steps in telomere replication. First, the telomere duplex is replicated resulting in either a blunt end (leading strand replication) or an overhang (lagging strand replication). The leading strand end is then processed to generate a G-overhang. Telomerase then extends the G-overhangs followed by C-strand fill-in to convert most of the ssDNA to duplex DNA, leaving a short G-overhang.

During S-phase, telomeres are replicated in three distinct steps (Figure 2C; Stewart et al., 2012). First, the duplex DNA is replicated by the conventional replication machinery. While replication on the leading strand is presumed to reach the chromosome terminus, the lagging strand machinery is unable to fully replicate the ends, a phenomenon known as the end-replication problem (Watson, 1972; Olovnikov, 1973). To overcome this, telomeres are extended by telomerase, which is recruited and stimulated by TPP1/POT1. Recent work suggests that TIN2 also mediates telomerase recruitment and functions with TPP1/POT1 to stimulate telomerase processivity (Frank et al., 2015; Pike et al., 2019). Prior to extension, telomeres are resected to create a binding site for telomerase. After extension, telomerase is then dissociated from the telomere by CTC1-STN1-TEN1 (CST), a replication protein A (RPA)-like ssDNA binding protein, to prevent extensive G-overhang elongation (Stewart et al., 2018; Lim and Cech, 2021). Both CST and RPA are heterotrimeric proteins that contain multiple ssDNA binding folds and recruit proteins to the DNA to perform various activities (Chen and Wold, 2014; Lim et al., 2020). Work in yeast also suggest that the Pif1 helicase may function to remove telomerase (Boule et al., 2005). CST is then proposed to stimulate DNA polymerase α-primase (pol α) to convert most of the G-overhang to duplex DNA (Giraud-Panis et al., 2010). The remaining short G-overhang can form a lariat structure called a telomere loop (t-loop) (Griffith et al., 1999). This structure is thought to protect the DNA terminus and restrict further access by telomerase, as discussed in more detail below. Telomeres can also be extended by a telomerase-independent mechanism that relies on recombination, a pathway known as alternative lengthening of telomeres (ALT) (Cesare and Reddel, 2010).

Together, telomerase and ALT make up the telomere maintenance pathways, which can coexist *in vivo* (Perrem et al., 2001). However, telomerase is the predominant elongation pathway under normal conditions. In humans, telomerase expression is typically restricted to germline and stem cells with most somatic cells having a finite number of cellular divisions. Once telomeres become critically short, cells lose the ability to divide, a state known as replicative senescence (Munoz-Espin and Serrano, 2014). Telomere shortening is associated with normal aging, and premature shortening is associated with a number of premature aging-related diseases (Armanios and Blackburn, 2012). A hallmark of cancer is replicative immortality; thus, pre-cancerous cells must maintain telomere length to prevent senescence (Hanahan and Weinberg, 2011). More specifically, 85 to 90% of human tumors re-express or upregulate telomerase while 10 to 15% maintain telomeres through ALT (Shay and Wright, 2019).

DSBs and telomeres resemble each other in many ways. Both are terminal DNA ends with a ssDNA overhang or blunt end. When such substrates arise in cells, decisions on whether or not to repair the DNA must be made. These decisions are often critical to maintaining genome stability with incorrect decisions potentially leading to cell death or chromosome instability. Accordingly, each decision point is highly regulated to ensure the proper repair pathway is engaged, or, in the case of chromosome ends, prevented. Many of these decision points are reversible, allowing a way back should the incorrect decision be made, or downstream factors are not available. However, the initial pathway choice often dictates the mechanism of repair. In this review, we will focus on these decision points and how they are regulated in mammals. Since HR-mediated DSB repair requires the most processing, it will be used as the focal point on which to frame decisions that direct pathway choice, including the mechanisms that shift repair toward HR vs. NHEJ and those protecting telomeres from “repair.”

## Mechanisms Regulating DSB Repair and End Protection

Based on current understanding, there are at least four key decision points required for HR-mediated DSB repair (Figure 3). First, the DNA ends are recognized and bound by the MRE11-RAD50-NBS1 (MRN) complex to initiate DNA repair and recruit the repair machinery. Second, the break is subjected to short-range resection by MRN. Third, long-range resection occurs to generate an overhang that is bound by RPA. Finally, RPA is replaced by RAD51, which formally initiates the homology search and HR-mediated repair. At each of these decision points, it is crucial to recognize whether the DNA end is a bona fide DSB vs. a chromosome terminus as well as whether a homologous sister chromatid is present. This will dictate how the DNA ends are processed and what factors are recruited. Below, we will broadly discuss each of these decision points and the factors regulating the choice to join or not join the DNA ends. For more detailed assessments of individual decisions points, we refer readers to several recent reviews (de Lange, 2018; Pannunzio et al., 2018; Wright et al., 2018; Krenning et al., 2019; Wu, 2019; Blackford and Stucki, 2020; Ensminger and Lobrich, 2020; Vitor et al., 2020; Yue et al., 2020; Panigrahi and Glover, 2021).

**FIGURE 3:** Key decision points in the repair of DSBs by HR. (1) The DNA ends are bound by either MRN or the Ku70/80 heterodimer. Binding and retention of MRN will shift repair toward HR and the binding of Ku shifts repair toward to NHEJ. (2) Short range resection by MRN. (3) Long-range resection of the DNA and RPA binding. (4) RPA is exchanged for RAD51, which facilitates strand invasion, DNA synthesis and HR repair.

### DSB Recognition

In response to DSBs, the lesion must first be recognized by DNA damage sensors. Ku binding is traditionally associated with repair by NHEJ whereas MRN is associated with HR-mediated repair. While still not completely understood, recent work, in both yeast and mammals, suggest that the recruitment and binding of these sensors is context dependent and not mutually exclusive (Langerak et al., 2011; Ingram et al., 2019; Chen et al., 2021). Instead, it is the subsequent steps that determine the displacement of these factors to promote HR, NHEJ or end protection. Recent biochemical and single molecule studies even suggest that Ku binding may be required for MRN-dependent resection (Deshpande et al., 2020). Much of this groundbreaking work has been performed in the model organism *S. cerevisiae* and then subsequently verified in mammals and other organisms. A major distinction between budding yeast and mammals is that NBS1 is not conserved in yeast. Instead, the *S. cerevisiae* complex is composed of Mre11, Rad50 and Xrs2 (MRX) with Xrs2 being the functional homolog of NBS1 (Rupnik et al., 2010; Tisi et al., 2020). For simplicity, we will use the designation MRN unless referring to studies exclusively performed in *S. cerevisiae*.

#### HR

MRN is one of the first responders to a DSB and, thus, it is key to instigating downstream steps in the repair process (Lisby et al., 2004). While recognition of the break by MRN is still under investigation, *in vitro* single molecule studies suggest that MRN uses facilitated 1D diffusion to search along nucleosome-bound DNA for DSBs (Myler et al., 2017). MRN can function at both unblocked and blocked DNA ends to promote resection of the DSB (Figure 4). At blocked ends, MRN can remove Ku as well as other protein-DNA adducts to access the break. MRN also promotes the recruitment and stimulation of ATM at the DSB, which in turn promotes H2AX phosphorylation on S139 (γH2AX) (Carney et al., 1998; Lee and Paull, 2004, 2005). Mediator of DNA damage checkpoint 1 (MDC1) is then recruited by γH2AX around the break and acts as a bridge between ATM and γH2AX to create a positive feedback loop (Burma et al., 2001; Kolas et al., 2007). Further expansion of γH2AX leads to the recruitment of additional downstream repair factors, the initiation of cell cycle arrest and resection of the DNA (Stewart et al., 2003; Stucki et al., 2005; Lou et al., 2006).

**FIGURE 4:** How DSB ends are processed under different conditions. Scissors indicate MRN endonuclease activity. MRN binding to unblocked ends leads to resection of the DNA. When Ku binds in the absence of MRN, no resection occurs. However, when both Ku and MRN are bound, stimulation of the MRN nuclease activity promotes resection and the removal of Ku. MRN can similarly function at ends blocked by a protein adduct, damaged bases or DNA secondary structures.

#### NHEJ

Like MRN, Ku is a first responder at DSBs and provides a docking site for DNA-PKcs (Yaneva et al., 1997). Unlike MRN, which can bind internally, Ku requires a free DNA end for binding and cannot associate with most blocked ends (Blier et al., 1993; Myler et al., 2017). Accordingly, when NHEJ is the preferred pathway, such as in G1, blocked ends must be freed to allow Ku binding (Mirman and de Lange, 2020). How these blocks are removed is still under investigation, but several nucleases, including tyrosyl-DNA phosphodiesterase 1 and 2 (TDP1/2) and Artemis, can remove hairpins, damaged bases or protein-DNA adducts (Menon and Povirk, 2016; Pannunzio et al., 2018; Meek, 2020). DNA blocks can also be removed through the stimulation of Artemis by DNA-PKcs (Gerodimos et al., 2017). Interestingly, in the event of a nucleosome blocked end, an *in vitro* study found that Ku can displace histone H1 from the DNA, however, it does not displace the nucleosome (Roberts and Ramsden, 2007). This could expose DNA ends to allow Ku binding, but more work is needed to uncover other possible roles of Ku in unblocking these DNA ends.

Whether Ku remains bound at the break appears to be one of the most critical steps in preventing resection and shifting repair outcomes toward NHEJ vs. HR. For Ku removal, several pathways can be employed to promote HR or, in the case of telomeres, end protection. These include the dissociation of Ku through short-range resection (discussed in more detail below), phosphorylation of Ku by DNA-PKcs, ubiquitination of Ku by RNF8 or RNF138 and blockage of DNA-PKcs autophosphorylation (Feng and Chen, 2012; Ismail et al., 2015; Lee et al., 2016). Autophosphorylation of DNA-PKcs is promoted through its interaction with the TIP60 histone acetyltransferase, which stimulate the activity of DNA-PKcs and recruitment of the ligation machinery (Ding et al., 2003). To block pro-NHEJ activity during S-phase, breast cancer gene 1 (BRCA1) directly blocks DNA-PKcs autophosphorylation (Davis et al., 2014). SUMOylation of TIP60 has also been proposed to inhibition autophosphorylation and facilitate a switch toward HR (Gao et al., 2020). Additionally, when homologous sequences are available during S and G2 phases, DNA-PKcs autophosphorylation favors the binding of MRN and other HR factors (Ding et al., 2003; Zhou and Paull, 2013; Symington, 2016). MRN can stimulate resection in the presence of Ku and DNA-PKcs through the recruitment of exonuclease 1 (EXO1) (Zhou and Paull, 2013). This allows the recruitment of EXO1 to DNA ends to promote HR rather than NHEJ, through mechanisms that are still poorly understood.

#### Telomeres

Although both Ku and MRN have been positively implicated in telomere maintenance (Wang et al., 2009; Lamarche et al., 2010), the exclusion of Ku and MRN from telomeres is one mechanism used to prevent the misrepair of chromosome ends. Mounting evidence indicates that t-loops serve a major role in blocking Ku and MRN access to chromosome ends (Figure 5). Recent analysis using super-resolution microscopy have helped define the mechanism of t-loop formation (Doksani et al., 2013; de Lange, 2018; Van Ly et al., 2018). This process is mediated by TRF2 and involves invasion by the G-overhang into duplex DNA to create a large lariat structure (Griffith et al., 1999; Doksani et al., 2013). While t-loops prevent initial recognition of telomeres as DSBs, these elegant structures must also be protected from the HR machinery. At the base of the t-loop, the DNA is presumed to form a Holliday junction (HJ)-like structure that can be cleaved by HJ resolvases, leading to telomere loss. Again, TRF2 is involved in preventing t-loop cleavage through inhibition of the Werner syndrome (WRN) helicase (Nora et al., 2010). This prevents WRN strand displacement of HJs with telomeric repeats (Nora et al., 2010). RAP1 has also been implicated in t-loop protection although some of the reports are conflicting (Bae and Baumann, 2007; Cesare et al., 2008; Benarroch-Popivker et al., 2016).

**FIGURE 5:** TRF2 facilitates telomere loop (t-loop) formation by promoting invasion of the G-overhang into the duplex region to form a displacement loop (D-loop). This t-loop combined with shelterin blocks MRN and Ku from accessing the chromosome ends and initiating DSB repair.

TRF2 deletion in mice results in removal of the 3′-ssDNA overhang by MRE11 and the loss of t-loops, promoting the “repair” of dysfunctional telomeres and chromosomal fusions (Attwooll et al., 2009; Deng et al., 2009; Cesare et al., 2013). When TRF2 is absent, ATM is phosphorylated in an MRN-dependent manner. However, the nuclease activity of MRE11 is dispensable, suggesting that MRN association alone is sufficient to recruit ATM to telomeres. Additionally, upon inhibition of TRF2, excision repair cross-complementation group 1 (ERCC1) and ERCC4 (also known as XPF) target the telomeric overhang for degradation (Zhu et al., 2003). This indicates a previously unexpected role of ERCC1/ERCC4 in the “repair” of unprotected telomeres through NHEJ. Interestingly, during G2, unprotected telomeres lacking a G-overhang are bound by Ku, which leads to chromosome fusions, although the DDR and formation of end-to-end fusions is functionally distinct from NHEJ (Zhu et al., 2003). In this case, RNF8 promotes the accumulation of ubiquitinated H2A, which in turn, recruits p53-binding protein 1 (53BP1), ATM and REV7 to promote DNA ligase IV-dependent NHEJ (Smogorzewska et al., 2002; Peuscher and Jacobs, 2011; Boersma et al., 2015).

### Short-Range Resection

Once a DSB is recognized by MRN, resection can be initiated to promote HR. This occurs in a two-step process with short-range resection by MRN followed by long-range resection to allow RPA-binding (Shibata et al., 2014). Once resection initiates, HR is enabled. This was previously seen as a point of no return. However, recent studies suggest that this decision point may be more flexible than initially imagined. Furthermore, resection is an essential step in telomere elongation so, under these conditions, resection needs to be achieved without engaging HR. In this section, the mechanisms regulating short-range resection will be discussed.

#### HR

Biochemical and single-molecule studies have significantly contributed to our understating of both short- and long-range resection in recent years. Combined with the many genetic studies performed in both yeast and mammals, the following model of short-range resection has emerged (Figure 6). First, MRE11 forms a nick in the dsDNA 20 to 40 nt from the break (Anand et al., 2016). Interaction between CtBP interacting protein (CtIP) (Sae2 in budding yeast) and MRN is essential for short-range resection (Huertas et al., 2008; Huertas and Jackson, 2009). MRE11 is a 3′-to-5′ exonuclease with weak endonuclease activity. Since resection creates a 3′-ssDNA overhang, it remained unclear for many years how resection was achieved through MRN. However, CtIP was discovered to stimulate the endonuclease activity of MRE11, allowing it to nick the dsDNA and create a template for MRN endonuclease activity (Anand et al., 2016). CtIP localization to DSBs is regulated by cyclin dependent kinase (CDK), BRCA1 and ATM (Yu and Chen, 2004; Yun and Hiom, 2009; Wang et al., 2013). In addition to regulating CtIP, CDKs also regulates other key factors involved in resection, checkpoint activation and downstream steps in the recombination process, making CDKs a vital player in pathway choice (Ferretti et al., 2013; Zhao et al., 2017). Since CDKs are cell cycle regulated, this helps prevent HR outside of S and G2 phase, which can have disastrous consequences.

**FIGURE 6:** Model of short-range resection. Short-range resection by MRN is stimulated by CtIP. Localization of CtIP to the chromatin is dependent on phosphorylation of CtIP by CDK and ATM and ubiquitination by BRCA1. CDK has also been proposed to phosphorylate MRX in budding yeast in a cell cycle-dependent manner, suggesting that CDK may regulate MRN in mammals. Phosphorylation of H2AX by ATM also promotes short-range resection and the recruitment of DSB machinery. Upon localization with MRN, CtIP stimulates both MRN endonuclease (indicated by the scissors) and 3′-to-5′ exonuclease activity to facilitate short-range resection. (P: phosphorylation; Ub: ubiquitination).

Stimulation of MRE11 nuclease activity may also be regulated by cell cycle and apoptosis regulator protein 2 (CCAR2) (Lopez-Saavedra et al., 2016). Work by López-Saavedra et al. suggests that MRN and CtIP are found in an inactive complex with CCAR2 and, upon DNA damage, phosphorylation of CtIP disrupts the CCAR2-CtIP-MRN complex to promote MRN nuclease activity. A complex of BRCA1 and BRCA1-associated RING domain-1 (BARD1) as well as exonuclease 3′-5′ domain-containing protein 2 (EXD2) also stimulate MRN-dependent nuclease activity and resection (Wang et al., 2007; Coleman and Greenberg, 2011; Broderick et al., 2016; Nieminuszczy et al., 2016). Recently, the lysine specific histone demethylase, PHF2 (KDM7C/JHDM1E), was shown to regulate CtIP and BRCA1 mRNA levels, suggesting an additional layer of regulation (Alonso-de Vega et al., 2020).

Once the nick is formed, MRE11 engages its 3′-to-5′ exonuclease activity to resect back toward the break (Shibata et al., 2014). This activity is also stimulated by CtIP, which is recruited by NBS1 (Wang et al., 2013; Anand et al., 2019). Additionally, the RAD50 subunit of MRN moderates MRE11 nuclease activity, indicating that MRN complex formation is critical to support short-range resection (Cannavo et al., 2019). The innerworkings of MRE11, RAD50 and NBS1 complex formation and activity has been well studied and reviewed extensively elsewhere (Lafrance-Vanasse et al., 2015; Reginato and Cejka, 2020; Qiu and Huang, 2021). Short-range resection by MRN is proposed to remove obstacles, such as Ku and other DNA adducts, freeing the DNA ends for repair by HR, alt-EJ or SSA (Figure 4; Chanut et al., 2016). In yeast, MRX works not only on blunt ends but also on chemically modified DNA, short overhangs and DNA containing secondary structures (Cejka, 2015).

#### NHEJ

Ku binding at DSBs serves as the major mechanism to block end resection (Rothkamm et al., 2003; Zhou and Paull, 2013; Ceccaldi et al., 2016; Graham et al., 2016; Mladenov et al., 2019). Accordingly, the decision to proceed toward NHEJ requires the prevention of MRN-dependent resection so that Ku remains bound. This can be achieved in several different ways. First, ATM limits resection by phosphorylating Ubiquilin 4 (UBQLN4), a proteasomal shuttle factor, which leads to MRE11 degradation (Jachimowicz et al., 2019). Thus, ATM plays seemingly contradictory roles in short-range resection. On the one hand, it promotes MRN-CtIP-BRCA1 recruitment to DSBs, while on the other, it promotes MRE11 degradation. Future work is needed to fully understand the role of ATM in DSB repair, but context (*e.g.*, cell cycle stage, location of the break, *etc.*) and the localization of other factors likely contribute to the use of ATM in NHEJ vs. HR. Another proposed mechanism to inhibit Ku removal is preventing MRN localization to the break site. While such a mechanism has not been directly demonstrated, cell cycle dependent phosphorylation of MRE11 by CDK1 was observed in *S. cerevisiae* and could serve to prevent MRE11 localization to DSBs (Simoneau et al., 2014). Once bound, MRN requires CtIP and other pro-resection factors to stimulate MRE11 nuclease activities. Thus, regulation of these factors can prevent resection and Ku removal. One strategy used to limit MRN nuclease activity is keeping CtIP levels low in G1 (Yu and Baer, 2000). Additionally, CtIP localization to DSBs is regulated by CDKs (CDK1 in yeast and CDK2 in mammals), as mentioned above. CDK-dependent phosphorylation of CtIP precipitates BRCA1 ubiquitination and CtIP localization to DSBs (Figure 6; Yun and Hiom, 2009; Wang et al., 2013). These modifications are mainly restricted to S/G2, limiting CtIP interaction with MRN. Interestingly, a recent report also found that long-term ATR kinase inhibition or conditional topoisomerase II binding protein 1 (TopBP1) degradation affects E2F-dependent transcription of BRCA1, CtIP and Bloom syndrome protein (BLM) (Dibitetto et al., 2020). Loss of these pro-resection factors results in impaired end resection and a shift toward toxic NHEJ, suggesting that translational regulation of pro-resection factors could also serve to regulate resection.

While NHEJ relies on the suppression of end resection for repair, in situations where NHEJ is impaired, alt-EJ and SSA works to join DSBs in a resection-dependent and Ku-independent manner (Figure 1; Ceccaldi et al., 2016). Generally, in these pathways, the DSB is first resected to expose ssDNA that varies in length depending on the pathway. In both pathways, MRN and CtIP initiate resection (Bennardo et al., 2008; Dinkelmann et al., 2009; Xie et al., 2009; Yun and Hiom, 2009; Zhang and Jasin, 2011; Truong et al., 2013; Biehs et al., 2017). If this initial end resection occurs in G1, it inhibits NHEJ and drives repair toward alt-EJ or SSA (Xiong et al., 2015; Bakr et al., 2016). Unlike HR, alt-EJ and SSA can repair DSBs during G1 of the cell cycle because a homologous sister chromatid is not required (Xiong et al., 2015; Sallmyr and Tomkinson, 2018). Alt-EJ is characterized by limited resection and short 2 to 20 nt regions of complementary sequences, while resection in SSA is longer and generally requires sequences of > 25 nt (Sallmyr and Tomkinson, 2018). After resection, the DNA ends are used to align short homologous sequences for repair. Non-homologous 3′ tails are then removed, gaps filled and the ends are ligated to complete repair (Figure 1).

#### Telomeres

During replication and telomere extension, telomeres are susceptible to recognition as DSBs and degradation. This is because the t-loop must be resolved to access the chromosome end (Figure 7). Furthermore, proteins involved in resection, including CtIP, EXO1 and DNA2, are involved in telomere duplex replication and could potentially act on chromosome ends (Lin et al., 2013; Stroik et al., 2019, 2020). On the leading strand, replication can theoretically proceed to the end of the chromosome to create a blunt end. This model is supported by studies in yeast, plants and mammals, where blunt-ends or very short (1 to 2 nt) overhangs have been identified after duplex replication (Chow et al., 2012; Valuchova et al., 2017). On the lagging strand, the RNA primer of the last Okazaki fragment must be removed, leading to a loss of at least 10 to 12 nt of DNA each replication cycle. However, analysis of G-overhangs suggests that the final Okazaki fragment actually initiates 70 to 100 nt from the chromosome terminus (Chow et al., 2012). Accordingly, the leading strand sister chromatid resembles a blunt-end or “clean” one-sided break whereas the lagging strand sister chromatid contains a significant ssDNA overhang, comparable to a resected DSB.

**FIGURE 7:** Model of telomere replication and end protection. During telomere replication, t-loops are resolved exposing chromosome ends to potential repair mechanisms. On the lagging strand, regions of ssDNA are bound by RPA as part of the normal replication process. To prevent stable RPA binding, an RPA-to-POT1 switch is facilitated by hnRNPA1. TERRA then removes hnRNPA1 to allow POT1 binding. On the leading strand, blunt telomere ends are resected by DNA2, EXO1 and/or Apollo to generate a G-overhang. (RPA may also bind to these ends and require removal). Telomerase is localized to the telomeres through its interaction with TPP1 to extend the G-overhang. To prevent G-overhang hyperextension, CST is localized to telomeres by TPP1 and inhibits telomerase activity. Additionally, CST promotes C-strand fill-in by stimulating pol α. After telomere processing, t-loops are reformed to protect the chromosome end from DSB repair.

In telomerase positive cells, the 3′-ssDNA overhang is extended in a highly controlled process to prevent potentially catastrophic events that may arise from telomere under- or over-extension. For extension by telomerase, a ssDNA binding site is needed to allow telomerase RNA component (TERC) to base pair, creating a primer for reverse transcription. While the lagging strand has a ready-made overhang, the leading strand requires processing. Studies in mice suggest that Apollo and EXO1 facilitate resection of the telomeric C-strand (van Overbeek and de Lange, 2006; Lam et al., 2010; Wu et al., 2010, 2012; Chow et al., 2012). In yeast, Dna2 has also been implicated in end processing, although it has been difficult to separate its role in duplex replication vs. end resection (Tomita et al., 2004; Budd and Campbell, 2013; Markiewicz-Potoczny et al., 2018). Currently, how Apollo, EXO1 and/or DNA2 are recruited for telomere end resection and whether the ends are immediately bound and protected by shelterin, following duplex replication, remains unclear. However, Apollo recruitment requires interaction with TRF2 and is subsequently blocked by POT1b (van Overbeek and de Lange, 2006; Wu et al., 2012). Therefore, shelterin, or at least shelterin subunits, are likely to bind immediately after passage of the replication fork, which could prevent recognition of the ends as DSBs.

T-loops are thought to serve as a major deterrent to HR and NHEJ. How t-loops are resolved to allow replication remains largely unknown but recent work by the Boulton group identified key steps in the assembly and disassembly process (Sarek et al., 2019). Outside of S-phase, t-loop formation is maintained by phosphorylation of TRF2 by CDK. During S-phase, TRF2 is transiently dephosphorylated by protein phosphatase 6 regulator subunit 3 (PP6R3), allowing t-loop disassembly and the completion of DNA replication. This t-loop disassembly appears to be very transient and another study suggests that t-loops may be present during S-phase (Timashev and De Lange, 2020). Thus, defining how this switch is regulated, and specifically how the DDR is inhibited during this period, warrants further investigation.

### Long-Range Resection

Short-range resection leads to additional processing to generate a long ssDNA overhang that becomes a substrate for RPA binding and the promotion of HR. The switch from short- to long-range resection, like other steps, is highly regulated and often described as a point of no return. However, as described in more detail below, mechanisms do exist to shift repair back to NHEJ, making this decision point reversible under certain conditions. Nevertheless, long-range resection and RPA binding are one of the most critical points in the pathway to joining DNA ends through HR vs. NHEJ. Moreover, telomeric G-overhangs must be protected from RPA binding and unwanted HR.

#### HR

The goal of long-range resection is to create a stretch of ssDNA long enough for significant RPA binding. RPA is then exchanged for RAD51, which facilitates the homology search. Critical to the initiation of long-range resection is the binding of BRCA1 and blockage of 53BP1 (Daley and Sung, 2014). Generation of the 3′-overhang by MRN likely leads to initial RPA binding and ATR recruitment. One model suggests an ATM to ATR switch in which ATM initiates resection and triggers ATR activation to regulate later steps in HR (Cuadrado et al., 2006; Shiotani and Zou, 2009). It is proposed that ATR drives HR by facilitating the stabilization of BRCA1 through TopBP1. This counteracts 53BP1 recruitment (Liu et al., 2017). BRCA1 and BARD1 then form a complex, which stabilizes BRCA1, to facilitate resection and recruit the partner and localizer of BRCA2 (PALB2)-BRCA2 complex for RAD51 loading (Joukov et al., 2006; Sy et al., 2009; Zhang et al., 2009b; Orthwein et al., 2015). The BRCA1-BARD1 complex also acts as an E3 ubiquitin ligase to prevent 53BP1 localization at DSBs during S phase (Chapman et al., 2012; Kakarougkas et al., 2013). While BRCA1 is not intrinsically required for resection, it is critical to overcome the 53BP1-mediated block and activation of DSB processing by facilitating CtIP phosphorylation (Cao et al., 2009; Bunting et al., 2010, 2012; Peterson et al., 2013; Nacson et al., 2018).

Long-range resection is primarily executed by two distinct pathways (Figure 8A; Nimonkar et al., 2011). The first involves EXO1, a 5′-to-3′ exonuclease (Tomimatsu et al., 2012; Myler et al., 2016). In this pathway, EXO1 enters at the 5′ site and generates an overhang several kilobases in length. *In vitro* biochemical assays have determined that EXO1 alone can perform end resection, although the process is slow (Soniat et al., 2019). Based on genetic and *in vitro* studies, MRN and the BLM helicase (Sgs1 in budding yeast) are proposed to recruit EXO1 and stimulate end resection (Mohaghegh et al., 2001; Nimonkar et al., 2011; Soniat et al., 2019). A second mechanism involves the joint effort of DNA2 and BLM. DNA2 is a structure-specific endonuclease that also possesses weak ATP-dependent helicase activity (Zheng et al., 2020). Since DNA2 does not possess exonuclease activity, the DNA is displaced into a flap structure for cleavage. Owing to the weak helicase activity of DNA2, current thinking, backed, by *in vitro* single-molecule studies, posits that BLM is required to create a 5′-DNA flap for cleavage (Mimitou and Symington, 2008; Nimonkar et al., 2011). Why two separate pathways exist is still unclear. However, recent biochemical reconstitution studies suggest that each may be tailored to deal with specific obstacles at or nearby the break site, such as ribonucleotides and DNA damage (Daley et al., 2020).

**FIGURE 8:** Models of long-range resection and how long-range resection is inhibited/reversed. **(A)** Long-range resection is mediated by EXO1 or BLM/DNA2. The resulting ssDNA is bound by RPA, which serves as a platform for ATR binding. To inhibit NHEJ, TopBP1 bridges interactions between ATR and the BRCA1-BARD1 complex, blocking 53BP1. **(B)** 53BP1 is localized to DSBs through its interaction with specific histone marks. 53BP1 then interacts with RIF1, which localizes the shieldin complex. Shieldin inhibits long-range resection by preventing access to the resected DNA and reverses resection through its interaction with CST-pol α, which can mediate fill-in of the resected DNA. This promotes repair of the break by NHEJ. (P: phosphorylation; Ub: ubiquitination).

CtIP and RPA have also been implicated as key stimulators of end resection. CDK phosphorylation of CtIP Thr847 is needed for effective ssDNA generation and RPA recruitment during long-range resection (Huertas and Jackson, 2009). *In vitro*, RPA stimulates BLM helicase activity at the nick created by MRN. However, phosphorylation of RPA70 inhibits DNA resection mediated by the BLM/EXO1 and BLM/DNA2 *in vitro* (Soniat et al., 2019; Qin et al., 2020). The dual roles of RPA in long range resection may explain how resection of the DNA is prevented while still promoting enough resection for HR.

#### NHEJ

To prevent long-range resection and promote NHEJ, genetic studies suggest that 53BP1 must outcompete BRCA1 for binding to MRN-generated overhangs (Setiaputra and Durocher, 2019). 53BP1 is localized to DSBs through its interaction with specific histone marks, including di-methylated histone H4 lysine 20 and ubiquitinated histone H2A lysine 15 (Figure 8B; Sanders et al., 2004; Botuyan et al., 2006; Kim et al., 2006; Yang et al., 2008; Hsiao and Mizzen, 2013). Upon localization to the DSB, 53BP1 works with various factors to prevent or reverse DSB resection. Pax2 transactivation domain interaction protein (PTIP) and Rap1-interacting protein 1 (RIF1) are two main factors downstream of 53BP1 which impair end resection at DSBs (Sfeir and de Lange, 2012; Zimmermann et al., 2013). PTIP acts by blocking DNA2 activity and interacts with the endonuclease Artemis to promote NHEJ (Wang et al., 2014; Callen et al., 2020). On the other hand, Rif1 limits the accumulation of BRCA1-BARD1 at DNA damage sites, preventing CtIP recruitment (Zimmermann et al., 2013).

The shieldin complex (SHLD1 [RINN3], SHLD2 [RINN2/FAM35A], SHLD3 [RINN1] and REV7 [MAD2L2/MAD2B]) also prevents and/or reverses end resection (Figure 8B; Setiaputra and Durocher, 2019). Shieldin was only recently discovered so many questions remain about how it functions in DSB repair. However, based on several mechanistic studies, a model has emerged in which shieldin both limits end resection and promotes the conversion of MRN-generated ssDNA back to duplex DNA. SHLD2 contains three predicted OB-folds that are proposed to bind to MRN-generated ssDNA overhangs, thus preventing long-range resection and RPA loading (Callen et al., 2020). To reverse end resection, shieldin recruits pol α and its stimulatory factor, CST (Mirman et al., 2018). CST/pol α then convert the ssDNA back to duplex DNA (Mirman et al., 2018; Noordermeer et al., 2018). How shieldin and CST/pol α are recruited to DSBs and under what circumstances is still not well understood. Nevertheless, recent studies suggest that TRIP13 and p31^*comet*^ promote HR by inactivating REV7, which could provide another reversal point back to HR (Clairmont et al., 2020; Sarangi et al., 2020). Another open question is whether 53BP1-shieldin-CST-pol α can act at DNA ends that escape initial 53BP1 binding and have already been resected. Such a mechanism could prevent the more disastrous effects of using alt-EJ or SSA rather than NHEJ in G1 (Ceccaldi et al., 2016). Shieldin can also act independently of 53BP1 to inhibit DSB resection, although the mechanism is still unclear (Ghezraoui et al., 2018). Future work on this newly discovered complex will undoubtedly uncover novel insight into this critical decision point.

#### Telomeres

Two key factors, POT1 and CST, are critical to prevent the recognition of telomeres as HR intermediates. In mammals, POT1 prevents RPA from binding the G-overhang, which in turn suppresses ATR activation and unwanted HR (Wu et al., 2006; Kratz and de Lange, 2018). Interestingly, studies in the protozoa *Leishmania amazonensis* and *Trypanosoma cruzi*, which appear to lack homologs of POT1 or CST, found that RPA-1 is involved in end protection, suggesting that under certain situations RPA can adapt telomere protection capabilities (Pavani et al., 2014, 2018; Fernandes et al., 2020). Since RPA has a higher binding affinity and is ∼70-fold more abundant, POT1 cannot outcompete RPA *in vitro* (Flynn et al., 2011; Hein et al., 2015). However, *in vivo* POT1 is tethered to shelterin through TPP1, giving POT1 a competitive advantage over RPA. Loss of TPP1 or the disruption of POT1/TPP1 and TIN2/TPP1 interaction results in telomeric RPA (Hockemeyer et al., 2007; Barrientos et al., 2008; Gong and de Lange, 2010; Kratz and de Lange, 2018). Additionally, POT1/TPP1 can protect uncapped telomeres following extensive resection, caused by the absence of TRF2 (Deng et al., 2009). During replication, however, shelterin is displaced and RPA binds to telomeres as part of the normal replication process (Figure 7). RPA must then be displaced for allow POT1 binding. Yet, POT1/TPP1 is unable to displace RPA from telomeric DNA *in vitro*. Instead, an elegant mechanism was uncovered in which RPA is displaced by heterogeneous nuclear ribonucleoprotein A1 (hnRNPA1) (Flynn et al., 2011; Figure 7). This RPA-to-POT1 switch is regulated in a cell cycle-dependent manner by expression of telomeric repeat-containing RNA (TERRA), a telomeric non-coding RNA.

Following replication, telomeres are extended in telomerase-positive cells. Under homeostatic conditions, telomerase adds ∼10 telomeric hexanucleotide repeats to each chromosome end and is then dissociated to prevent excessive G-overhang lengthening (Zhao et al., 2009, 2011). Termination of telomerase activity is primarily mediated by CST (Chen et al., 2012). The PIF1 helicase can also remove telomerase, although it is unclear whether this function is solely used to prevent *de novo* telomere addition at DSBs or can also promote telomerase dissociation from telomeres under certain conditions (Boule et al., 2005; Zhang et al., 2006; Churikov and Geli, 2017). Removal of telomerase is critical for end protection, as hyper-extension of G-overhangs can result in telomeric RPA due to the exhaustion of available POT1 (Feng et al., 2017, 2018). While still not completely understood, mammalian CST is thought to localize to telomeres through interactions with TPP1/POT1 (Wan et al., 2009; Chen et al., 2012). TPP1/POT1 also recruits telomerase so a switch likely occurs where telomerase is replaced by CST. A similar mechanism of overhang processing has been extensively studied in *S. cerevisiae*. Since shelterin is not present in *S. cerevisiae*, Cdc13 recruits telomerase for telomere extension and Stn1-Ten1 for C-strand fill-in, in place of TPP1/POT1 (Tseng et al., 2006; Li et al., 2009; Shen et al., 2014; Gopalakrishnan et al., 2017). This process is regulated by a series of post-translational modifications. In humans, phosphorylation of TPP1 by NIMA related kinase 6 (NEK6) is proposed to facilitate telomerase recruitment but much of the mechanism remains unknown (Zhang et al., 2013; Hirai et al., 2016). Furthermore, how CST is recruited to telomeres, whether its recruitment displaces telomerase from TPP1 and the role of CST DNA binding activity in this process remain open questions.

In addition to inhibiting telomerase, CST promotes C-strand fill-in by stimulating pol α (Stewart et al., 2018). CST regulated fill-in does not appear to be as critical as its ability to modulate telomerase inhibition for end protection. Deletion of human TEN1 resulted in defective C-strand fill-in but CTC1-STN1 were still able to inhibit telomerase. This led to only a minor increase in G-overhang elongation and the absence of RPA binding, suggesting that under these conditions POT1 levels were sufficient to block RPA (Feng et al., 2018). Similar results were obtained with knockdown of CST subunits (Surovtseva et al., 2009; Wang et al., 2012; Kasbek et al., 2013). Interestingly, analysis of G-overhangs across the cell cycle in STN1 knockdown cells showed that elongated G-overhangs were reset to near wild-type levels upon entry into the next G1 (Wang et al., 2012). The mechanism behind this reset is unknown but may be due to low levels of STN1 that promote fill-in of the overhang in G2 or M phase. It is also possible that backup mechanisms exist to rescue lingering, elongated G-overhangs and prevent potential RPA binding.

### RPA-to-RAD51 Exchange

Following long-range resection, RPA is exchanged for RAD51 to promote the homology search for HR repair. The homologous template is then used to fill-in the missing sequence for error-free repair of the DSB. The switch to RAD51 is generally thought to be an irreversible step toward HR over NHEJ. However, there is new evidence that even at this late stage, mechanisms may be in place to prevent HR under specific situations. At telomeres, the best way to prevent HR is preventing RPA binding, but what happens to G-overhangs that become stably bound by RPA? Below, we will discuss regulation of the RPA-to-RAD51 switch at DSBs and telomeres as well as how ALT is used to extend telomeres but prevent end joining.

#### HR

After resection, ssDNA is quickly bound by RPA. For HR-mediated repair, RPA is replaced with RAD51 to form a RAD51-ssDNA nucleoprotein filament, also known as the presynaptic complex (Lee et al., 2015; Qi et al., 2015). *In vitro* single-molecule studies of RPA and RAD51 exchange indicated that although RPA binds to ssDNA with a higher affinity than RAD51, high concentrations of RAD51 can undergo facilitated exchange following ATP hydrolysis by RAD51 (Ma et al., 2017). However, *in vivo* RAD51 mediator proteins facilitate the binding, elongating, and stabilization of RAD51 onto ssDNA. BRCA2 is primarily responsible for delivering RAD51 monomers (Wong et al., 1997; Pellegrini et al., 2002; Esashi et al., 2007; Carreira et al., 2009; Jensen et al., 2010). BRC repeats in BRCA2 act as a scaffold to bind RAD51, a process facilitated by BRCA1 and PALB2. PALB2 bridges the interaction between BRCA1 and BRCA2 and localizes RAD51 to the RPA-ssDNA, where RAD51 is exchanged for RPA (Scully et al., 1997; Xia et al., 2006; Sy et al., 2009; Zhang et al., 2009a, b; Zong et al., 2019). After RAD51 filament formation, RAD51 paralogs aid in stabilization and elongation of the filament (Thacker, 1999; Suwaki et al., 2011; Sullivan and Bernstein, 2018). While filament formation is essential for HR, the exchange of RAD51 for RPA can be detrimental at other sites of RPA-ssDNA in the cell, such as replication forks. To prevent these untimely exchanges, RPA1-related ssDNA binding protein, X-linked (RADX) was found to antagonize RAD51-ssDNA filament formation, inhibiting RPA displacement as well as promoting the disassembly of existing RAD51 filaments at stalled replication forks (Zhang et al., 2020). Once formed, RAD51 filaments search for homologous regions in the sister chromatid to instigate repair, as reviewed in detail elsewhere (Haber, 2018; Bonilla et al., 2020).

Although most studies have focused on 53BP1 function prior to DSB resection, recent data in budding yeast raises the possibility that 53BP1 functions after long-range resection and RPA binding. The 53BP1 homolog Rad9 was shown to promote D-loop extension by limiting Sgs1 (BLM in mammals) and Mph1 (FANCM in mammals) helicase activity, suggesting a role in HR sub-pathway choice after DSB end resection (Ferrari et al., 2020). The proposed model is that after a DSB, Rad9 limits hyper-loading of RPA, Rad51, and Rad52. This limits Sgs1 and Mph1 from strand rejection to facilitate long-lived D-loops, thus favoring repair through sub-pathways that require stable D-loops such as break induced replication (BIR) or long tract gene conversion. If strand rejection occurs, then SSA is favored. This unprecedented role of Rad9 in controlling the fate of HR contradicts the commonly thought of role of 53BP1 in DSB repair, where it acts as a pre-resection block to HR in eukaryotes. Whether 53BP1 functions in the same manner in humans is still unclear, but it could have paradigm-shifting implications for 53BP1 activity at later steps in DSB repair, if true.

#### Telomeres

In the majority of cancers, telomeres are maintained in a telomerase-dependent manner, however, 10 to 15% of human cancers maintain their telomeres through the use of ALT (Bryan et al., 1997). ALT is a homology-based mechanism to lengthen telomeres (Dunham et al., 2000; Hoang and O’Sullivan, 2020; Recagni et al., 2020; Sommer and Royle, 2020; Zhang and Zou, 2020). The mechanisms of ALT are still under investigation, but recent evidence points to ALT using a BIR-like mechanism, which requires the exchange of RPA to induce recombination (Dilley et al., 2016). ALT is characterized by ALT-associated promyelocytic leukemia (PML) bodies (APBs), which consist of telomeric DNA, PML, and proteins involved in DNA repair, recombination and replication (Zhang and Zou, 2020). It is still not fully understood how APBs are assembled and how they promote ALT. However, a model has been proposed where BLM is critical for APB formation and telomeric DNA synthesis (Stavropoulos et al., 2002; Zhang et al., 2019). Additionally, MRN is localized to telomeres during S and G2 phases through its interaction with TRF2 and is required for ALT (Zhu et al., 2000; Jiang et al., 2005; Zhong et al., 2007). Within the APBs, the telomere is lengthened through RAD51- or RAD52-dependent BIR-like pathways. In both cases, a homology search is utilized to initiate BIR. In the RAD51-dependent pathway, RAD51 and HOP2-MND1 are recruited, and then RAD51 mediates homology searches and subsequent DNA polymerization (Cho et al., 2014). In RAD52-dependent BIR, BLM and DNA2 are proposed to resect the telomere and then replication factor C (RFC) mediates proliferating cell nuclear antigen (PCNA) loading (Dilley et al., 2016). PCNA recruits pol δ through interaction with POLD3 stimulating pol δ activity and DNA synthesis (Dilley et al., 2016; Roumelioti et al., 2016). Thus, for ALT, the engagement of BIR-related factors vs. those required for HR-mediated repair appears to underlie telomere extension while preventing chromosome fusions.

As described above, preventing stable binding and localization of HR factors is the major mechanism used to prevent unwanted “repair” at telomeres, but what happens when RPA remains stably bound to G-overhangs? Loss of POT1 or CST results in telomeric RPA foci but surprisingly only a minor increase in chromosome fusions, particularly in comparison to TRF2 loss (Denchi and de Lange, 2007; Feng et al., 2017). Once bound by RPA, telomeres, in essence, resemble resected RPA-bound DSB intermediates. Even in the absence of POT1, other shelterin subunits are present and likely play a role in maintaining end protection. Yet, how these RPA-bound telomeres remain protected from HR is not entirely clear. It is likely that the presence of 53BP1 contributes to protection from HR. 53BP1 foci have been observed at telomeres in both cells lacking POT1 (Hockemeyer et al., 2007; Gong and de Lange, 2010) and cells expressing a CTC1 G503R mutant construct, which is unable to localize to telomeres (Chen et al., 2013; Gu and Chang, 2013; Takai et al., 2016). In both cases, hyper-extended G-overhangs are generated. Under such conditions, 53BP1 may continue to block HR, while TRF2 is used to block NHEJ (Figure 9). In addition, deletion of CTC1 decreases TopBP1 and CHK1 phosphorylation, despite RPA-binding and ATR activation at telomeres (Ackerson et al., 2020). The loss of CHK1 signaling and 53BP1 localization could be sufficient to block the RPA-to-RAD51 exchange and, thus, HR-mediated telomere fusions at RPA-bound telomeres. However, additional studies are needed to determine the fate of RPA-bound telomeres. Unraveling such mechanism(s) will undoubtedly provide novel insights into chromosome end protection and HR-mediated repair.

**FIGURE 9:** Potential mechanism for the protection of RPA-bound telomeres. Loss of POT1 or CST results in hyperextension of G-overhangs and telomeric RPA but very few fusions events. We propose that the combination of TRF2 and 53BP1 prevent fusions by blocking NHEJ and HR mediated repair, respectively.

## Conclusion

While our understanding of DSB recognition and repair has progressed by leaps and bounds in recent years, important questions remain unanswered. Two key topics that still need to be fully elucidated are the context and timing of the key decision points described in this review. To date, much of our current understanding has centered on how specific factors interact with each other. To grasp the larger picture, we must now understand the temporal and contextual organization of these processes. This includes addressing how and when t-loops are formed, when shelterin disassembly/reassembly occurs and elucidating the mechanisms that protect exposed ends. Furthermore, understanding DSB pathway choice will require addressing questions such as the timing of Ku vs. MRN binding at DSBs, whether MRN is removed in situations where a homologous sequence is unavailable and how stimulation of MRN nuclease activities are temporally regulated. Such advances will pave the way for a more mechanistic understanding of these complex processes. Finally, both dysfunctional DSB repair and telomeres are linked to cancer and aging-related diseases. Therefore, defining the decision points that dictate whether to join or not to join the DNA ends will enlighten how these diseases arise and uncover vulnerabilities that might be exploited for therapeutic purposes.

## Author Contributions

SA designed the graphics. All authors wrote and edited the manuscript, contributed to the article and approved the submitted version.

## Conflict of Interest

The authors declare that the research was conducted in the absence of any commercial or financial relationships that could be construed as a potential conflict of interest.
